The article "Solving an Infectious Disease Model considering Its Anatomical Variables with Stochastic Numerical Procedures" was published in 2022. Journal: J Healthc Eng.

# Solving an Infectious Disease Model considering Its Anatomical Variables with Stochastic Numerical Procedures

**DOI:** 10.1155/2022/3774123

**Published:** 2022-01-07

**Authors:** Zulqurnain Sabir, Muhammad Asif Zahoor Raja, Yolanda Guerrero Sánchez

**Affiliations:** ^1^Department of Mathematics and Statistics, Hazara University, Mansehra, Pakistan; ^2^Future Technology Research Center, National Yunlin University of Science and Technology, 123 University Road, Section 3, Douliou, Yunlin 64002, Taiwan; ^3^Department of Anathomy and Pscicobiology, Faculty of Medicine, University of Murcia, Murcia 30100, Spain

## Abstract

The aim of the current work is to perform the numerical investigation of the infectious disease based on the nonlinear fractional order prey-predator model using the Levenberg–Marquardt backpropagation (LMB) based on the artificial neuron networks (ANNs), i.e., LMBNNs. The fractional prey-predator model is classified into three categories, the densities of the susceptible, infected prey, and predator populations. The statistics proportions for solving three different variations of the infectious disease based on the fractional prey-predator model are designated for training 80% and 10% for both validation and testing. The numerical actions are performed using the LMBNNs to solve the infectious disease based on the fractional prey-predator model, and comparison is performed using the database Adams–Bashforth–Moulton approach. The infectious disease based on the fractional prey-predator model is solved using the LMBNNs to reduce the mean square error (M.S.E). In order to validate the exactness, capability, consistency, and competence of the proposed LMBNNs, the numerical procedures using the correlation, M.S.E, regression, and error histograms are drawn.

## 1. Introduction

Infectious diseases occur when some viruses, fungi, germs, and parasites enter into the human body. These forms are diffused through infection from one to another human, contaminated food, animals, or contact to any of the ecological factors that are polluted with any type of these bodies. Every infection-based disease has its own symptoms, types, and severity. A few common symptoms of these infections in the body include pain, flu, cough, and fever [1, 2]. Some of the infections have minor symptoms that do not need any cure or treatment. Alternatively, there are various serious deathly cases that may disturb the population equilibrium of numerous classes in the atmosphere. For the last few years, mathematical systems are used to predict the species evolution. It initiated from the Lotka and Volterra systems [3, 4], where their expediency in evading several worst situations for many species as death was evidenced. Currently, researchers apply this tool to reveal the consequence of a certain policy used by some of the governments to handle few species that can be measured as a significant device to preserve each kind.

The article "Solving an Infectious Disease Model considering Its Anatomical Variables with Stochastic Numerical Procedures" was published in 2022. Journal: J Healthc Eng.

The ecological systems are more complex for any type of infection, which can affect the growth of few classes, as a personification. In this study, a predator-prey collaboration is considered. This contagion may distress the predator strength and the hunting competence that takes few of the predators in the position of death. In the previous studies, numerous investigations have examined the predator-prey interactions in the occurrence of transmittable viruses; see, for instance, [5, 6] where predator-prey models are treated with an analytical approach, while in [7–9], these models have a numerical analysis. As an alternative, there are various approaches, which reflect the predators to accomplish an effective hunt. The hunting collaboration is one of the operating policies of the predator, where numerous predators work to hunt some prey. This scheme is valuable to reduce the rate of hunting, and a number of hunters behave in this technique. The high rate of efficiency is seen in hunting lions, wild dogs, and hyenas. The mathematical system of this precise predator behavior was modeled and presented for the first time in [10], in which a simple model was applied to describe a cooperation. So far, there have been a few studies of the predator-prey interaction behavior presented in these references: in [11], the hunting effect is considered, in [12], the cooperation effect is considered, in [13], hunting and cooperation effects are considerd at the same time, and finally, in [14], hunting and cooperation effects are considered jointly with the Alle effect. Therefore, it has investigated the effects of a transmittable virus in the predator-prey communication along with the occurrence of the collaboration of predator hunting.

A three-species system is considered an infection in a prey population, which is categorized into two classes, the infected and susceptible prey. It is found that the derivative forms of time fractional have widespread applications to describe various forms of actual conditions that are recognized by the memory outcomes of a dynamical form. The memory rate is known as the derivative order, and the function of memory is called the fractional-order derivative. The time-fractional derivative is implemented to model the phenomena of various real-world problems [15, 16]. The nonlinear fractional-order prey-predator model has three classes, mathematically written as follows [17]:

(1) $$\begin{array}{c} \left\{\begin{array}{cc} D^{\alpha }S\left(\tau \right)=r\left(I\left(\tau \right)+S\left(\tau \right)\right)-\left(aP\left(\tau \right)+\lambda \right)P\left(\tau \right)S\left(\tau \right)-\delta S\left(\tau \right)I\left(\tau \right)-\mu S\left(\tau \right), & S\left(0\right)=k_{1},\\ D^{\alpha }I\left(\tau \right)=\delta I\left(\tau \right)S\left(\tau \right)-\left(\text{aP}\left(\tau \right)+\lambda \right)P\left(\tau \right)I\left(\tau \right)-\mu I\left(\tau \right), & I\left(0\right)=k_{2},\\ D^{\alpha }P\left(\tau \right)=e\left(\text{aP}\left(\tau \right)+\lambda \right)P\left(\tau \right)\left(I\left(\tau \right)+S\left(\tau \right)\right)-\text{mP}\left(\tau \right), & P\left(0\right)=k_{3}, \end{array}\right) \end{array}$$

where *S*(*τ*) and *I*(*τ*) are the densities of the susceptible and infected prey, while *P*(*τ*) shows the densities of predator populations. The term *e* signifies the rate of conversion of prey into predator biomass (susceptible or infected). The parameter *r* represents the prey population's reproduction number, and it is supposed that this infection does not convey vertically. It can also be defined as mother-child, where the predator is not diseased by this virus after a direct interaction with the diseased prey. The rate of transmission of the prey population, i.e., infection rate, is represented by *δ*. The functional form (aP(*τ*)+*λ*)*P*(*τ*)*S*(*τ*) and (aP(*τ*)+*λ*)*P*(*τ*)*I*(*τ*) are the hunting cooperation values [10]. The death rate of the population of the prey is *μ*, which represents the natural mortality rate of the predator's population. The initial conditions are *k*_1_, *k*_2_, and *k*_3_, respectively.

The article "Solving an Infectious Disease Model considering Its Anatomical Variables with Stochastic Numerical Procedures" was published in 2022. Journal: J Healthc Eng.

The aim of the current work is to perform the numerical investigation of the infectious disease based on the fractional prey-predator model using the Levenberg–Marquardt backpropagation (LMB) based on the artificial neuron networks (ANNs), i.e., LMBNNs. The LMBNNs are applied on three different variants of authentication, testing, training, and sample information. The statistics proportions for solving three different variations of the infectious disease based on the fractional prey-predator model are designated for training 80% and 10% for both validation and testing. The numerical results are performed using the LMBNNs to solve the infectious disease based on the fractional prey-predator model, and comparison is performed using the database Adams–Bashforth–Moulton approach. Recently, the stochastic computing solvers are applied based on the heuristic and swarming techniques in frequently reported articles of utmost significance [18–21]. However, the infectious disease spread systems governed with the fractional prey-predator model have never implemented to study its solution dynamics by using the competency of LMBNNs' computing paradigm. A few novel features and contribution of the current investigations are provided in brief as follows:

- The design of stochastic computing solvers LMBNNs is presented for the first time to solve the infectious disease spread systems governed with the fractional prey-predator model
- The designed procedures of LMBNNs have been implemented effectively to study the behavior of different scenarios of the fractional prey-predator model, and comparative studies are found in decent resemblance with the state-of-the-art Adams–Bashforth–Moulton numerical approach for solving fractional differential equations
- The convergence performances on iterative updated of MSE, negligible absolute error (AE) from standard outcomes, correlation/regression index, and error histograms (EHs) further authenticate the efficacy of the designed LMBNN computing platform for fractional prey-predator models

The paper is organized as follows: Section 2 shows the methodology based on LMBNNs.  Section 3 presents the numerical outcomes through LMBNNs to solve the fractional-order nonlinear prey-predator model. The final comments are reported in Section 4.

The article "Solving an Infectious Disease Model considering Its Anatomical Variables with Stochastic Numerical Procedures" was published in 2022. Journal: J Healthc Eng.

## 2. Methodology: LMBNNs

In this section, the proposed methodology of LMBNNs is presented for the infectious disease based on the fractional-order nonlinear prey-predator system. The methodology is categorized in two steps. The necessary trials of the stochastic-based LMBNNs are provided, and the execution process of the stochastic computing scheme is given to solve the infectious disease based on the nonlinear fractional-order prey-predator model.

A suitable optimization procedure-based proposed LMBNN is plotted in Figure 1 together with the outcomes and analysis of the results, while for a single neuron, the designed procedure is given in Figure 2. The stochastic computing-based procedures are executed using the “nftool” (MATLAB build-in command in the neural networks toolbox). The dataset for the fractional-order nonlinear prey-predator system is designated for training 80% and 10% for both validation and testing in LMBNN operations.

## 3. Numerical Procedures of the Fractional-Order Nonlinear Prey-Predator System

The current section shows the numerical procedures of the infectious disease based on the fractional-order nonlinear prey-predator system by applying the proposed computing stochastic LMBNNs. The literature parameter forms to solve the infectious disease based on the nonlinear fractional-order prey-predator model are *r*=1.5, *λ*=0.5, *a*=0.5, *δ*=0.5, *μ*=0.5, *e*=0.5, *m*=0.5, *k*_1_=0.2, *k*_2_=0.7, and *k*_3_=0.6. Three cases using the variations of fractional-order derivative, i.e., *α*  = 0.5, 0.7, and 0.9, are provided to solve the infectious disease based on the fractional-order nonlinear prey-predator system. The inclusive results have been performed for each category of the fractional-order nonlinear prey-predator system which are in between [0, 1] with 0.01 step size. Ten numbers of neurons throughout this numerical study have been taken, and the data are designated for training 80% and 10% for both validation and testing. The achieved numerical values using the LMBNNs to solve the infectious disease based on the fractional-order nonlinear prey-predator system are drawn in Figure 3. The representations based on the LMBNNs to solve the infectious disease based on the fractional prey-predator system are given in Figures 4–8. The M.S.E measures and state transitions (STs) to solve the infectious disease based on the fractional prey-predator model are plotted in Figure 4. The M.S.E based on the training, states of best curves, authentication, and testing is drawn in Figures 4(a)–4(c)), whereas the best ST values to solve the fractional prey-predator model are derived in Figures 4(d)–4(f)) at epochs 325, 387, and 127, respectively. The obtained performances exist around 1.3399 × 10^−10^, 1.4672 × 10^−10^, and 5.2351 × 10^−10^, respectively. The gradient performances of the LMBNNs to solve the infectious disease based on the fractional prey-predator model are found around 8.0331 × 10^−06^, 9.9161 × 10^−08^, and 9.8524 × 10^−08^, respectively. These calculated performances plotted in the figures show the accuracy, convergence, and precision of the proposed stochastic procedures of the LMBNNs to solve the infectious disease based on the fractional prey-predator model. The plots of the fitting curves to solve the fractional prey-predator model are given in Figures 5(a)–5(c)), which show the comparative analysis of the obtained outcomes through LMBNNs.  Figure 5(d)–5(f)) show the values of the EHs that exists around 6.63 × 10^−07^, 8.31 × 10^−06^, and 3.19 × 10^−05^ for the 1^st^, 2^nd^, and 3^rd^ case, respectively. The values of the regression are drawn in Figures 6–8 to solve the infectious disease based on the fractional prey-predator model. These illustrations of the correlations indicate regression soundings found around 1 that authenticates the perfect model. The testing, verification, and training plots designate the exactness of the LMBNNs to solve the infectious disease based on the fractional prey-predator model. In addition, the convergence performances through M.S.E based on the epochs, training, complexity, testing, backpropagation performances, and verification are provided in Table 1 to solve the infectious disease based on the nonlinear fractional prey-predator model.

The article "Solving an Infectious Disease Model considering Its Anatomical Variables with Stochastic Numerical Procedures" was published in 2022. Journal: J Healthc Eng.

The comparative performances and the AE values are illustrated in Figures 9 and 10 for the fractional prey-predator model. The outcomes for each category of the fractional prey-predator system presented using the stochastic LMBNNs are given in Figures 9(a)–9(c)). The matching of the obtained and reference solutions for each category of the infectious disease is perceived based on the fractional-order nonlinear prey-predator model. These outcomes matching represent the accurateness of the stochastic LMBNNs for each category of the infectious disease based on the fractional order nonlinear prey-predator system, The AE measures for each category of the infectious disease based on the fractional-order nonlinear prey-predator system are plotted in Figures 10(a)–10(c)). The AE for *S*(*τ*) based on the fractional-order nonlinear prey-predator system is calculated around 10^−04^ to 10^−06^ for case 1 and 3, while the AE is calculated 10^−05^ to 10^−06^ for case 3. The AE for *I*(*τ*) based on the fractional-order nonlinear prey-predator model is calculated around 10^−04^ to 10^−07^ for case 1, 10^−05^ to 10^−09^ for case 2, and 10^−05^ to 10^−07^ for case 3. The AE for *P*(*τ*) based on the fractional-order nonlinear prey-predator model is calculated around 10^−05^ to 10^−08^ for case each case of the nonlinear system.

## 4. Conclusions

In these investigations, the solutions of an infectious virus based on the nonlinear fractional prey-predator system are numerically presented by using the stochastic procedures based on the Levenberg–Marquardt backpropagation along with artificial neural networks. These stochastic-based procedures LMBNNs are provided to solve three cases by taking different values of the fractional order. The numerical solutions have been performed using the sample data, testing, training, and authentication. The data proportions to solve the nonlinear fractional prey-predator model are designated for training 80% and 10% for both validation and testing. The numerical results of the infectious disease based on the nonlinear fractional prey-predator model are achieved using the LMBNNs, and comparison is performed using the database Adams–Bashforth–Moulton approach. The solutions of the fractional-order nonlinear model are obtained through the LMBNNs in order to reduce the M.S.E. To indorse the exactness, capability, dependability, and competence of the proposed LMBNNs, the numerical procedures are provided using the M.S.E, correlation, EHS, and regression. The matching of the results designates the precision of the designed scheme, and the values of the AE in good ranges for each case of the infectious disease based on the nonlinear fractional prey-predator model show the effectiveness of the scheme.

The article "Solving an Infectious Disease Model considering Its Anatomical Variables with Stochastic Numerical Procedures" was published in 2022. Journal: J Healthc Eng.

In future, the procedures based on the LMBNNs are applied to get the outcomes of the fractional-order systems and Lonngren-wave systems [22–26]. Additionally, one may exploit the Bayesian regularization method-based neural networks for solving different scenarios of the fractional prey-predator model for better outcomes in terms of accuracy and efficiency.

## Figures and Tables

**Figure 1:** Workflow illustration of the designed LMBNNs to solve the infectious disease based on the nonlinear fractional prey-predator model.

**Figure 2:** Proposed framework using a single neuron.

**Figure 3:** Proposed LMBNN to solve the infectious disease based on the nonlinear fractional prey-predator model.

**Figure 4:** M.S.E measures (a–c) and ST performances (d–f) to solve the infectious disease based on the fractional prey-predator model. (a) Case 1: M.S.E. (b) Case 2: M.S.E. (c) Case 3: M.S.E. (d) Case I: EHs. (e) Case 2: EHs. (f) Case 3: EHs.

**Figure 5:** Result assessments (a–c) and EHs (d–f) to solve the infectious disease based on the fractional prey-predator model. (a) Case 1: result assessments. (b) Case 2: result assessments, (c) Case 3: result assessments. (d) Case I: EHs. (e) Case 2: EHs. (f) Case 3: EHs.

**Figure 6:** Regression measures of the fractional-order nonlinear prey-predator model of case 1.

**Figure 7:** Regression measures of the fractional-order nonlinear prey-predator model of case 2.

**Figure 8:** Regression measures of the fractional-order nonlinear prey-predator model of case 3.

**Figure 9:** Comparison illustrations to solve the infectious disease based on the nonlinear fractional prey-predator model. (a) Results for *S*(*τ*). (b) Results for *I*(*τ*). (c) Results for *P*(*τ*).

**Figure 10:** AE values to solve the infectious disease based on the nonlinear fractional prey-predator model. (a) AE for *S*(*τ*). (b) AE for *I*(*τ*). (c) AE for *P*(*τ*).

**Table 1:** Statistical measures to solve the infectious disease based on the nonlinear fractional prey-predator model.

Case	M.S.E for samples in			Performance	Gradient	Mu	Epoch	Time
	Training	Validation	Testing					
1	3.21 × 10^−09^	1.33 × 10^−10^	2.29 × 10^−09^	2.63 × 10^−09^	8.03 × 10^−06^	1.00 × 10^−10^	325	5
2	2.43 × 10^−10^	1.46 × 10^−10^	5.44 × 10^−10^	2.43 × 10^−10^	9.92 × 10^−08^	1.00 × 10^−10^	387	5
3	4.63 × 10^−10^	5.23 × 10^−10^	2.19 × 10^−08^	4.63 × 10^−10^	9.85 × 10^−08^	1.00 × 10^−09^	127	2

## Data Availability

No data were used to support this study.
